# Clinical Observation of Laser Peripheral Iridoplasty with Number of Laser Shots in the Treatment of Acute Angle-Closure Glaucoma

This article has been retracted.

**DOI:** 10.1155/2022/7968999

**Published:** 2022-03-15

**Authors:** Cheng Ma, Zengye Liu, Wei Zhao, Luning Hei, Shuang Yao

**Affiliations:** Department of Ophthalmology, Tianjin First Central Hospital, School of Medicine, Nankai University, Tianjin 300192, China

## Abstract

**Objective:**

To quantitatively study the intraocular pressure (IOP) control and chamber angle opening degree of patients with acute angle-closure glaucoma (stage of attack) treated by laser peripheral iridoplasty (LPIP) with different numbers of laser shots, and to evaluate the efficacy and safety of different numbers of laser shots.

**Methods:**

Fifty-five patients (60 eyes) with acute angle-closure glaucoma treated in our hospital from May 2019 to December 2020 were selected as the research subjects. All patients had poor intraocular pressure control (≥40 mmHg) after IOP-lowering drug therapy. The patients were randomly divided into three groups, 20 eyes in each group, and underwent laser peripheral iridoplasty (LPIP) with different numbers of laser shots (group I: 35 laser shots, group II: 45 laser shots, and group III: 60 laser shots). The best-corrected visual acuity, IOP, corneal condition, and opening degree of anterior chamber angle (ACA), namely, the trabecular-iris angle (TIA), angle opening distance at 500 *μ*m (AOD_500_), and complications of patients before LPIP, 2 hours after LPIP, and 24 hours after LPIP were observed, and the opening degree of ACA were quantitatively measured.

**Results:**

The corrected visual acuity of the three groups after LPIP was improved to varying degrees, and the IOP decreased, TIA and AOD_500_ were increased compared with those before operation, and the differences were statistically significant (*P* < 0.05). There were statistically significant differences between group II and group I (*P* < 0.05). Four eyes in group I underwent LPIP again due to increased IOP. In group III, iris hemorrhage occurred in one eye and iris depigmentation occurred in one eye, and there was no statistical difference compared with group II (*P* > 0.05).

**Conclusions:**

LPIP can effectively reduce preoperative IOP and increase ACA width in patients with persistent high IOP that failed to respond to drug therapy, and moderate numbers of laser shots can achieve satisfactory results and highest safety.

## 1. Introduction

Glaucoma is a progressive optic neuropathy having specific pattern of visual field defects and characteristic appearances of the optic discs. It is classified into open‐angle or closed‐angle glaucoma based on appearance of anterior chamber angle. An elevated intraocular pressure (IOP) is built as a result of the obstruction of the outflow pathway located in the anterior chamber angle by peripheral iris [1, 2]. Many individuals with appositional anterior chamber angle closure have normal IOP and no glaucoma symptoms. They have “narrow angles” or “primary angle closure suspects” (PACs). If the IOP is high and/or there is synechial closure (but no glaucomatous damage), the phrase “primary angle closure” (PAC) is recommended. Primary angle-closure glaucoma (PACG) is defined as angle closure with glaucomatous optic disc injury and/or visual field loss. Angle closure refers to patients with narrow angles, PAC, or PACG [1]. Glaucoma is the main cause of permanent blindness worldwide. Glaucoma affects 67 million individuals globally. PACG is more prevalent than OAG, although it is more likely to cause bilateral blindness [3, 4]. The disease affects Asians and women more than Caucasians [5]. In China, Foster et al. found 28.2 million people have narrow angles [6], whereas 9.1 million have closed angles [7]. Moreover, PACG causes 91 percent of the 1.7 million bilaterally blinded Chinese glaucoma patients. PACG may be the main cause of glaucoma blindness today, according to Foster and Johnson [8].

The acute attack of primary acute angle-closure glaucoma is an ocular emergency. If it is not treated in time and effectively, the optic nerve will be irreversibly damaged, which will greatly affect the prognosis of vision [9]. Clinically, many patients cannot effectively control intraocular pressure (IOP) even with the combined use of topical and systemic IOP-lowering drugs. For many years, laser iridoplasty can successfully open the angle-closure glaucoma [10]. Laser peripheral iridoplasty (LPIP) can reduce IOP effectively by photocoagulation of iris root to make iris tissue shrink and open the angle of the chamber to increase the outflow of aqueous humor. In this study, the postoperative effects of LPIP with different numbers of laser shots were observed in three groups of patients, and the appropriate number of laser shots was explored to obtain the best therapeutic effect and maximum safety.

## 2. Materials and Methods

### 2.1. General Information

From May 2019 to December 2020, 55 patients (60 eyes) with acute primary acute angle-closure glaucoma who were admitted to our department and emergency department for outpatient, emergency, and inpatient treatment and whose IOP still could not be controlled after IOP-lowering drugs were selected. There were 21 males (22 eyes) and 34 females (38 eyes), aged from 55 to 72 years, with an average of 63.4 years.

### 2.2. Inclusion Criteria

Patients with an onset time of 12–72 hours, all had been treated with local or systemic IOP-lowering drugs for 1–3 days, and the IOP was not well controlled (≥40 mmHg) were included in the study. No IOP-lowering drugs were used before onset. There was no other primary disease in the eye and no history of eye surgery.

### 2.3. Methods

The affected eyes were randomly divided into three groups, with 20 eyes in each group; all LPIP were completed by the same doctor who was proficient in LPIP. The three groups were respectively applied with different numbers of laser shots, with 35 in group I, 45 in group II, and 60 in group III. The patients were treated with the Sitron 532 laser produced by LUMENIS Medical Laser Company. Half an hour before the operation, 1% pilocarpine eye drops were given to reduce pupil, and proparacaine hydrochloride eye drops were used for topical anesthesia. After the iris microscope was placed, 360° photocoagulation was performed on the iris root with spot diameter of 300 *μ*m, energy of 180–200 mw, and exposure time of 0.2–0.4 s. After operation, pranoprofen eye drops and fluorometholone eye drops were given.

### 2.4. Observation Indicators

The best-corrected visual acuity, corneal condition, and opening degree of anterior chamber angle (ACA), namely, the trabecular-iris angle (TIA), angle opening distance at 500 *μ*m (AOD500), and complications of the three groups of patients before LPIP, 2 hours after LPIP, and 24 hours after LPIP were observed. The IOP changes were measured with a noncontact tonometer, and the opening degree of ACA was quantified by OCT.

### 2.5. Statistical Methods

Statistical software SPSS (version 22.0) was used to analyze the data. Completely random grouping design was adopted. The data of all indicators were expressed as‾mean ± standard deviation (*x* ± *s*). One-way ANOVA was used to compare the difference in decrease of IOP, increase of degree of TIA, and increase of distance of TOD_500_ among the three groups at each time point. If there were differences, the LSD-T test was used for further pairwise comparison between the three groups. *P* < 0.05 was considered statistically significant.

## 3. Results

### 3.1. The Distribution of Best-Corrected Visual Acuity before and after Surgery in the Three Groups of Patients

The best-corrected visual acuity of the three groups of patients before surgery was less than 0.5, which was improved to varying degrees after surgery (Table 1).

### 3.2. The IOP of the Three Groups of Patients

The average preoperative IOP of patients in the three groups were 55.4 ± 10.2 mmHg, 57.7 ± 7.6 mmHg, and 56.2 ± 8.3 mmHg, respectively; the average IOP 2 hours after the operation were 20.3 ± 5.6 mmHg, 17.2 ± 6.3 mmHg, and 18.9 ± 4.9 mmHg, respectively; the average IOP 24 hours after surgery were 19.2 ± 8.3 mmHg, 17.9 ± 4.9 mmHg, and 17.6 ± 8.4 mmHg, respectively (Table 2, Figure 1).

### 3.3. TIA of the Three Groups of Patients

The average preoperative TIA of the three groups of patients were 7.4 ± 3.2°, 7.7 ± 5.4°, and 7.2 ± 4.3°, respectively; the average TIA 2 hours after operation were 23.3 ± 4.1°, 25.2 ± 2.3°, and 26.9 ± 4.6°, respectively; the average TIA 24 hours after operation was 25.2 ± 3.8°, 27.3 ± 4.7°, and 27.6 ± 8.2°, respectively (Table 3).

### 3.4. TOD_500_ of the Three Groups of Patients

The average preoperative TOD_500_ of the three groups of patients were 105 ± 064 *μ*m, 114 ± 054 *μ*m, and 109 ± 043 *μ*m, respectively; the average TOD_500_ 2 hours after surgery were 273 ± 041 *μ*m, 325 ± 083 *μ*m, and 330 ± 046 *μ*m, respectively; the average TOD_500_ 24 hours after surgery were 285 ± 110 *μ*m, 331 ± 050 *μ*m, and 329 ± 042 *μ*m, respectively (Table 4, Figure 2).

### 3.5. Comparison of Postoperative Changes in IOP, TIA, and TOD_500_ among the Three Groups

The changes in IOP, TIA, and TOD_500_ were compared among the three groups. The results showed that there were differences among the three groups (*P* < 0.05), the increase degree of TIA and TOD_500_ in group II and III was significantly higher than that in group I (*P* < 0.05), while there was no statistically significant difference between group II and group III (*P* > 0.05) (Table 5).

### 3.6. Intraoperative and Postoperative Complications and Treatment

In group I, four eyes were treated with LPIP again due to increased IOP, and postoperative IOP was controlled. The IOP in group II was well controlled, and no abnormal condition was found. In group III, iris depigmentation was observed in one eye after the operation, IOP was normal, and no special treatment was given except local application of pranoprofen eye drops and fluorometholone eye drops. In group III, one eye had iris hemorrhage after operation, and Zhikang capsule was given orally for 3 days. The hematocele was absorbed, and the IOP was normal (Figure 3).

## 4. Discussion

With the aging of the population, glaucoma is still the first irreversible blinding eye disease in the world [11]. Therefore, timely and effective control of IOP and maintenance of stable target IOP value is of great importance. The occurrence of angle-closure glaucoma is closely related to the anatomy of anterior segment of the eyeball and the state of the lens. Short ocular axis, shallow anterior chamber, narrow chamber angle, thick lens, and its anterior position are all predisposition factors. In addition to the traditional pupillary block factors, there are still a variety of nonpupil block factors, including peripheral iris accumulation, anterior position of the ciliary body, and anterior displacement of lens. In acute onset of acute angle-closure glaucoma, the sudden closure of ACA causes a sharp increase in IOP. If the IOP is not controlled in time, it will cause irreversible damage to the optic nerve. Therefore, early and rapid reduction of IOP is very important for patients with acute attack.

The traditional treatment method for acute angle-closure glaucoma in acute attack stage is local application of IOP-lowering drugs, combined with systemic application of hypertonic agents and carbonic anhydrase inhibitors, and the IOP of most patients can be effectively controlled [12]. However, for some patients and some patients with cardiac and renal insufficiency who cannot use hypertonic agents, the IOP is often not effectively controlled. Although anterior chamber puncture and discharge can temporarily reduce IOP, the stable IOP-lowering effect cannot be maintained due to the continuous closure of ACA. Due to severe corneal edema and extremely shallow anterior chamber during acute attack, peripheral iridotomy is not the best treatment method. Besides, trabeculectomy under high IOP is a risky operation, which is prone to serious complications such as malignant glaucoma and explosive suprachoroidal hemorrhage during and after operation. Therefore, it is necessary to seek an effective and safe treatment to reduce IOP before glaucoma filtration surgery.

In previous reports, laser treatment is mostly LPIP, but it mainly relieves angle-closure glaucoma caused by pupillary block factors and has no obvious effect on angle-closure glaucoma caused by other factors [5, 13]. LPIP has become one of the important methods for the treatment of acute angle-closure glaucoma in recent years and has been widely used in clinical practice. LPIP is applied to the peripheral iris by laser photocoagulation, which causes the iris matrix to shrink, mechanically pulls open the ACA, reopens the closed ACA, and increases aqueous humor outflow [14]. Although the laser operation is simple and convenient, it can quickly open the ACA and reduce the IOP, but the unreasonable laser energy and exposure time can produce complications such as corneal injury, aggravation of anterior chamber inflammation, iris hemorrhage or atrophy, and pupil dilation. Therefore, it is our focus to explore the reasonable numbers of laser shots and obtain the most effective and safe therapeutic effect through the minimum laser energy, that is, the minimum damage.

Previous studies mostly observed the effectiveness of LPIP surgery, but there was no report on how much total laser energy could achieve the best therapeutic effect with the highest safety and minimum complications. In this study, the basic parameters of laser treatment, namely, spot diameter, single laser energy, and action time were relatively fixed, and the number of laser shots was set as a variable. Also, the number of laser shots from 35 to 60 was selected through clinical experience and the subjects were divided into three groups (group I: 35 laser shots, group II: 45 laser shots, and group III: 60 laser shots). The results showed that IOP in all three groups decreased at 2 and 24 hours after surgery, and TIA and TOD_500_ increased at different degrees compared with before surgery. Compared with group I, IOP decreased significantly in group II and group III, and the opening degree of ACA increased, the difference was statistically significant. Four eyes in group I underwent LPIP again due to increased IOP, and postoperative IOP was controlled. This suggested that with the increase of the number of laser shots, that is, the total laser energy, the decrease in IOP increased, and the opening degree of ACA increased, and the treatment effect was obvious. However, there was no statistically significant difference between group III and group II. In addition, with the increase in number of laser shots from 45 to 60, one eye had iris depigmentation and one eye had iris hemorrhage after surgery, suggesting that the opening degree of ACA will not increase infinitely after the increase in number of laser shots, and there will be complications related to laser treatment in the eye. Therefore, moderate laser shots, that is, the total laser energy of about 45 laser shots, is safer, more effective, and has less side effects.

## 5. Conclusion

In conclusion, LPIP should be actively performed for patients with acute angle-closure glaucoma who are ineffective in local and systemic drug treatment. The moderate laser shots, that is, about 45 laser shots, can effectively reduce IOP, which is safe and effective, creating opportunities for glaucoma surgery and avoiding the risk of glaucoma filtration surgery under high IOP. However, the number of cases observed in this study was limited, and trabeculectomy was performed in some patients within one week after LPIP, and the observation time was only 24 hours after LPIP. Therefore, long-term clinical observation with large samples is still needed for the observation of long-term effect of LPIP.

## Figures and Tables

**Figure 1:** Comparison of preoperative and postoperative IOP among the three groups.

**Figure 2:** (a, b) TIA (ACA) at 3 o'clock and 9 o'clock before LPIP were 8° and 9°, respectively, and TOD_500_ were 143 *μ*m and 153 *μ*m, respectively; (c, d) TIA (ACA) at 3 o'clock and 9 o'clock after LPIP were 23° and 25°, respectively, and TOD_500_ were 358 *μ*m and 487 *μ*m, respectively; suggesting that TIA (ACA) and TOD_500_ increased after LPIP compared with before surgery.

**Figure 3:** (a, b) appearance of the right eye and left eye at the attack stage of acute angle-closure glaucoma after treatment with IOP-lowering drugs, showing ciliary hyperemia, corneal edema, and slightly dilated pupil.

**Table 1:** The distribution of best-corrected visual acuity before and after surgery in the three groups of patients (number of eyes).

Time point	Group I			Group II			Group III		
	＜0.1	0.1–0.5	＞0.5	＜0.1	0.1–0.5	＞0.5	＜0.1	0.1–0.5	＞0.5
Before surgery	15	5	0	13	7	0	14	6	0
2 hours after surgery	2	8	12	0	4	16	0	5	15
24 hours after surgery	2	7	11	0	3	17	0	4	16

**Table 2:** Preoperative and postoperative IOP of patients in the three groups (mmHg) ($\bar{x}$ ± *s*).

Time point	Different numbers of laser shots		
	Group I (30–40)	Group II (40–50)	Group III (＞60)
Before surgery	55.4 ± 10.2	57.7 ± 7.6	56.2 ± 8.3
2 hours after surgery	20.3 ± 5.6	17.2 ± 6.3	18.9 ± 4.9
24 hours after surgery	19.2 ± 8.3	17.9 ± 4.9	17.6 ± 8.4

**Table 3:** Preoperative and postoperative ACA opening degree of three groups of patients (°) ($\bar{x}$ ± *s*).

Different numbers of laser shots			
Time point	Group I (30–40)	Group II (40–50)	Group III (＞60)
Before surgery	7.4 ± 3.2	7.7 ± 5.4	7.2 ± 4.3
2 hours after surgery	18.3 ± 4.1	21.2 ± 2.3	22.9 ± 4.6
24 hours after surgery	20.2 ± 3.8	23.3 ± 4.7	24.6 ± 8.2

**Table 4:** Preoperative and postoperative TOD_500_ of the three groups (*μ*m) ($\bar{x}$ ± *s*).

Different numbers of laser shots			
Time point	Group I (30–40)	Group II (40–50)	Group III (＞60)
Before surgery	105 ± 064	114 ± 054	109 ± 043
2 hours after surgery	273 ± 041	325 ± 083	330 ± 046
24 hours after surgery	285 ± 110	331 ± 050	329 ± 042

**Table 5:** Changes in IOP, TIA, and TOD_500_ were compared among the three groups.

Group	Decrease in IOP (mmHg)		Increase in TIA (°)		Increase in TOD_500_ (*μ*m)	
	2 hours after surgery	24 hours after surgery	2 hours after surgery	24 hours after surgery	2 hours after surgery	24 hours after surgery
Group I	34.9 ± 5.3	35.9 ± 4.6	12.2 ± 5.6	13.2 ± 3.6	181 ± 064	202 ± 106
Group II	38.6 ± 5.9	37.9 ± 4.8	15.2 ± 8.1	16.3 ± 4.8	223 ± 012	252 ± 129
Group III	38.8 ± 7.4	38.1 ± 6.1	16.9 ± 3.4	17.1 ± 2.2	243 ± 105	256 ± 047

F	4.512	3.462	5.101	4.547	3.689	5.478
*P* value	＜0.05	＜0.05	＜0.05	＜0.05	＜0.05	＜0.05
t group I vs. group II	9.105	10.231	8.342	7.115	7.412	6.532
*P* value group I vs. group II	＜0.05	＜0.05	＜0.05	＜0.05	＜0.05	＜0.05
t group I vs. group III	8.143	7.450	9.145	8.542	6.543	8.141
*P* value group I vs. group III	＜0.05	＜0.05	＜0.05	＜0.05	＜0.05	＜0.05
t group II vs III	0.356	0.245	1.435	0.657	1.230	0.856
*P* value group II vs III	＞0.05	＞0.05	＞0.05	＞0.05	＞0.05	＞0.05

## Data Availability

The data will be available from the corresponding author upon request.
